# Central Exercise Action Increases the AMPK and mTOR Response to Leptin

This article has been retracted.

**DOI:** 10.1371/journal.pone.0003856

**Published:** 2008-12-04

**Authors:** Eduardo R. Ropelle, Maria Fernanda A. Fernandes, Marcelo B. S. Flores, Mirian Ueno, Silvana Rocco, Rodrigo Marin, Dennys E. Cintra, Lício A. Velloso, Kleber G. Franchini, Mario J. A. Saad, José B. C. Carvalheira

**Affiliations:** Department of Internal Medicine, FCM, State University of Campinas (UNICAMP), Campinas, São Paulo, Brazil; University of Las Palmas de Gran Canaria, Spain

## Abstract

AMP-activated protein kinase (AMPK) and mammalian Target of Rapamycin (mTOR) are key regulators of cellular energy balance and of the effects of leptin on food intake. Acute exercise is associated with increased sensitivity to the effects of leptin on food intake in an IL-6-dependent manner. To determine whether exercise ameliorates the AMPK and mTOR response to leptin in the hypothalamus in an IL-6-dependent manner, rats performed two 3-h exercise bouts, separated by one 45-min rest period. Intracerebroventricular IL-6 infusion reduced food intake and pretreatment with AMPK activators and mTOR inhibitor prevented IL-6-induced anorexia. Activators of AMPK and fasting increased food intake in control rats to a greater extent than that observed in exercised ones, whereas inhibitor of AMPK had the opposite effect. Furthermore, the reduction of AMPK and ACC phosphorylation and increase in phosphorylation of proteins involved in mTOR signal transduction, observed in the hypothalamus after leptin infusion, were more pronounced in both lean and diet-induced obesity rats after acute exercise. Treatment with leptin reduced food intake in exercised rats that were pretreated with vehicle, although no increase in responsiveness to leptin-induced anorexia after pretreatment with anti-IL6 antibody, AICAR or Rapamycin was detected. Thus, the effects of leptin on the AMPK/mTOR pathway, potentiated by acute exercise, may contribute to appetite suppressive actions in the hypothalamus.

## Introduction

Prolonged exercise of medium to high intensity is known to profoundly affect energy balance [1]–[3]. Studies of individuals who have maintained significant weight loss for >1 year have demonstrated that dieters who achieve long-term success are often those who engage in regular and extensive exercise programs [4]. Although the energy expenditure aspects of such exercise may contribute to the effects of weight maintenance, it has been suggested that exercise may also contribute to the energy balance by altering food intake [5], [6]. Rodents submitted to exercise have increased sensitivity to leptin, conversely animals with diet-induced obesity and most obese humans are resistant to leptin [5], [7], [8]. Thus, the mechanism for leptin increased responsiveness in exercise is of great interest and understanding this mechanism could lead to new approaches to prevent or treat obesity.

The hypothalamus plays a central role in integrating hormonal (leptin and insulin) and nutritional signals from the periphery and modulating food intake, energy expenditure, and peripheral metabolism [9]. Multiple factors control food intake, including hormones, fuels and behaviour. AMPK is the downstream component of a kinase cascade that acts as a sensor of cellular energy charge, being activated by rising AMP coupled with falling ATP. Once activated, AMPK phosphorylates acetyl-CoA carboxylase (ACC) and switches on energy-producing pathways at the expense of energy-depleting processes [10]–[12]. Another target molecule for the control of food intake and energy homeostasis is represented by the phosphoprotein mammalian target of rapamycin, mTOR, in which the PI(3)K/Akt pathway has been suggested to affect the mTOR phosphorylation state and catalytic activity [13]. Activated signaling through mTOR phosphorylates the serine/threonine kinase p70S6K and the translational repressor eukaryotic initiation factor (eIF) 4E binding protein (4EBP1) [14], [15]. mTOR signaling is inhibited under conditions of low nutrients, such as glucose and amino acids and low intracellular ATP levels [16]. While mTOR was presumed to serve as the direct cellular sensor for ATP levels [17], mounting evidence has implicated AMPK in the regulation of mTOR activity [15], [18]–[20].

The level of circulating interleukin-6 (IL-6) increases dramatically in response to exercise [21], with IL-6 being produced by working muscle [22], [23] and adipose tissue [24], [25] and its concentration correlates temporally with increases in AMPK in multiple tissues [26]. In addition, AMPK activity is diminished in IL-6 deficient mice at rest and the absolute increases in AMPK activity in these tissues caused by exercise is diminished compared with control mice [27]. It also appears that centrally-acting IL-6 plays a role in the regulation of appetite, energy expenditure, and body composition [5], [28]. The signaling mechanism of IL-6 in the hypothalamus is, however, not fully understood. In cells, binding IL-6 to the α subunit of its receptor triggers the recruitment of gp130, subsequently leading to the activation of the gp130-associated JAK [29]–[31]. JAK links cytokine receptor to the STAT3 and MAP kinase pathway [29], [30], [32]. In addition to JAK/STAT and MAP kinase pathways, IL-6 also activates the PI(3)K/Akt pathway [33].

In this study, we sought to determine whether the improved response of the AMPK and mTOR pathways to leptin could contribute to the increased molecular response of leptin in rats submitted to exercise in an IL-6-dependent manner. We therefore, examined hypothalamic modulation of AMPK/ACC and mTOR signaling pathways, induced by IL-6, as well as the role of IL-6 in those signaling pathways induced by leptin in rats after acute exercise.

## Results

### IL-6 decreases hypothalamic AMPK and increases mTOR signaling

To determine whether IL-6 modulates hypothalamic AMPK/ACC signaling, we injected IL-6 into the third ventricle of rats and evaluated food intake and AMPK signaling. IL-6 caused a significant reduction in food intake (Figure 1a). We next investigated whether the microinfusion of IL-6 modulates the hypothalamic ATP concentration. Figure 1b shows that IL-6 (200 ng) changed ATP, ADP and AMP concentrations in the hypothalamus of rats, whereas, sixty minutes after IL-6 injection, the ATP content increased by ∼88% (Figure 1c) and decreased AMP∶ATP ratio by ∼54% in Wistar rats (Figure 1d). Consistent with the modulation of the AMP∶ATP ratio, we observed reduced hypothalamic AMPK and ACC phosphorylation induced by IL-6 (Figures 1e and f); whilst IL-6 increases p70S6K and 4EBP1 phosphorylation (Figures 1g and h). The αAMPK, ACC, p70S6K and 4EBP1 protein levels were not different between the groups (Figures 1e–h, lower panels).

**Figure 1:** Effects of IL-6 on food intake, hypothalamic AMPK/mTOR activity and ATP content. (a) Effect of i.c.v. administration of IL-6 on food intake; pretreatment with AICAR blocks IL-6-induced anorexia (*n* = 12–15 animals per group). (b, c, d) Typical chromatographic run (b) depicting the ATP, ADP, and AMP fractions in control (black line) and in i.c.v. IL-6 treated animals (red line), as mean ATP content and as AMP∶ATP ratio (c, d). (e, f, g, h) Representative Western blots of four independent experiments showing hypothalamic lysates from Wistar rats. Phospho-AMPK^thr172^, threonine-phosphorylated AMPK and total AMPK (e); phospho-ACC^ser79^, serine phosphorylated ACC and total ACC (f); phospho-p70S6Kinase^thr389^, threonine phosphorylated p70S6Kinase and total p70S6K (g); phospho-4EBP1^thr70^, threonine phosphorylated 4EBP1 and total 4EBP1 (h). Confocal microscopy was performed using IL-6 receptor (IL-6R)-specific antibody (green) and DAPI (blue), with 50× magnification (i). Co-localization of IL-6R (green) and AMPK (red) and IL-6R (green) and phospho-p70S6K (red) 60 minutes after i.c.v. saline or IL-6 infusion in the arcuate nuclei of rats, with 200× magnification (j). Data are the means±SEM. *p<0.05, *vs.* control group; **p<0.01, *vs.* control group; # *p*<0.05, *vs.* other groups.

If the effect of IL-6 on food intake is mediated by AMPK inhibition, AICAR infusion at doses that do not change food intake, but still increase AMPK and ACC phosphorylation, could be sufficient to block the effects of IL-6. Thus, to determine whether the effects of IL-6 on food intake are AMPK-dependent, we first identified a dose of AICAR that did not alter food intake (0.5 mM) when administered at the onset of the dark cycle. We then evaluated the effect of i.c.v. pretreatment with this dose of AICAR, or its vehicle, on the anorectic response to i.c.v. IL-6 (200 ng) and we observed that the anorectic response to i.c.v. IL-6 was reversed by AICAR at the time points studied (figure 1a). These findings indicate that inactivation of neuronal AMPK is necessary for some of the effects of IL-6 on food intake.

Immunohistochemistry with anti-Interleukin-6 Receptor (IL-6R)-specific antibody showed that IL-6R is expressed in a majority of neurons in the arcuate nucleus (Figure 1i). Double-staining confocal microscopy showed the positive immunoreactivity of IL-6R and AMPK in the hypothalamic arcuate nucleus of rats 60 minutes after i.c.v. saline or IL-6 (200 ng) infusion. The immunoreactivity of IL-6R and pp70S6K was not detected in the hypothalamic arcuate nucleus of rats after i.c.v. saline infusion. However, we observed the positive double-staining of IL-6R and pp70S6K 60 minutes after i.c.v. IL-6 (200 ng) infusion (Figure 1j).

### IL-6 induction of hypothalamic mTOR does not require changes in PI(3)K signaling

If the effect of IL-6 on food intake is mediated by mTOR activation, Rapamycin infusion at doses that do not change food intake, but still decrease p70S6K and 4EBP1 phosphorylations could be sufficient to block the effects of IL-6. Thus to determine whether IL-6 modulates hypothalamic mTOR signaling, we injected IL-6 (200 ng) into the third ventricle of rats and evaluated food intake and mTOR signaling. IL-6 caused a significant reduction in food intake (Figure 2a) and induced hypothalamic p70S6K and 4EBP1 phosphorylation (Figures 2b and c). The p70S6K and 4EBP1 protein levels were not different between the groups (Figures 2b and c, lower panels). To determine whether the effects of IL-6 on food intake are mTOR-dependent, we first identified a dose of Rapamycin that did not alter food intake (25 µg) when administered at the onset of the dark cycle. We then evaluated the effect of i.c.v. pretreatment with this dose of Rapamycin or its vehicle, on the anorectic response to i.c.v. IL-6 and we observed that IL-6 reduction of food intake was reversed by Rapamycin.

**Figure 2:** Effects of IL-6 on food intake and hypothalamic PI(3)K/mTOR and JAK/STAT activity. (a) Pretreatment with Rapamycin blocks IL-6-induced anorexia (*n* = 10–12 animals per group). (b, c) Representative Western blots of four independent experiments showing hypothalamic lysates from Wistar rats. Phospho-p70S6Kinase^thr389^, threonine phosphorylated p70S6Kinase and total p70S6K (b); phospho-4EBP1^thr70^, threonine phosphorylated 4EBP1 and total 4EBP1 (c). (d) Pretreatment with LY294002 had no effect on anorectic response to IL-6 (*n* = 10–12). (e) Representative western blot of four independent experiments showing hypothalamic lysates from Wistar rats. Phospho-Akt^ser473^, serine phosphorylated Akt and total Akt. (f) Pretreatment with AG490 blocks IL-6-induced anorexia (*n* = 10–12 animals per group). (g, h) Representative Western blots of four independent experiments showing hypothalamic lysates from Wistar rats. Phospho-JAK2, tyrosine phosphorylated JAK2 and total JAK2 (g); phospho-STAT3, Tyrosine phosphorylated STAT3 and total STAT3 (h). Data are the means±SEM. **p<0.01, *vs.* control group; # *p*<0.05, *vs.* other groups.

We next examined whether PI(3)K signaling is required for the IL-6-dependent reduction of food intake, by IL-6 administration in LY294002 pretreated (i.c.v.) animals. Pretreatment with LY294002 at a dose that did not alter food intake (1 nmol) had no effect on anorectic response to i.c.v. IL-6 (Figure 2d). Consistent with these data, we observed that a single IL-6 i.c.v. injection did not change Akt phosphorylation status in the hypothalamus (Figure 2e). The Akt protein levels were not different between the groups (Figure 2e, lower panel). These findings indicates that activation of neuronal mTOR is necessary for some of the effects of IL-6 on food intake and that these effects of IL-6 do not require any change in PI(3)K signaling.

We also injected IL-6 (200 ng) into the third ventricle of rats and evaluated food intake and JAK2/STAT3 signaling. IL-6 caused a significant reduction in food intake (Figure 2f) and induced hypothalamic JAK2 and STAT3 phosphorylation (Figures 2g and h). The JAK2 and STAT3 protein levels were not different between the groups (Figures 2g and h, lower panels). To determine whether the effects of IL-6 on food intake are also JAK2/STAT3-dependent, we first identified a dose of AG490 that did not alter food intake when administered at the onset of the dark cycle. We then evaluated the effect of i.c.v. pretreatment with this dose of AG490 or its vehicle, on the anorectic response to i.c.v. IL-6 and we observed that IL-6 reduction of food intake was reversed by AG490 (Figure 2f).

### Physiological parameters measured in basal conditions after exercise protocol

The plasma glucose level was lower in the exercised group compared to the control group (3.6±0.8 *vs* 4.6±0.5 mmol/L; n = 5; *p*<0.05) and the insulin levels were also lower (88±12 *vs* 193±17 pmol/L, n = 5; *p*<0.05). Exercise did not, however, reduce plasma leptin (2.6±0.5 *vs* 2.3±0.7 ng/ml). Insulinemia and leptinemia were not altered by third ventricle microinjection of leptin (data not shown).

### Exercise partially reverses the effects of AMPK agonists and fasting on food intake through modulation of the AMPK-mTOR signaling pathway in the hypothalamus

To test the role of a single session of exercise on AICAR-increased food intake, AICAR (2 mM) or its vehicle were administered (i.c.v.) to control and exercised animals. 12-hour total food intake was measured after exercise. In exercised rats, AICAR (2 mM) did not cause any acute change in food intake but, in the control group, AICAR (2 mM) increased food intake by 32% (Figure 3a), suggesting that AICAR is not effective in exercised rats. Comparing AICAR-treated groups (control *vs.* exercise), exercised animals showed a 33% reduction in 12-hour total food intake (Figure 3a).

**Figure 3:** AICAR, 2-DG and fasting effects on 12-h cumulative food intake and AMPK/mTOR signaling, in the hypothalami of control and exercised rats. (a) AICAR (2 mM) was administered in control and exercised rats. Animals were immediately exposed to food for a 12-hour period (*n* = 12–15 animals per group). (b, c, d, e) Representative Western blots of five independent experiments showing hypothalamic lysates from Wistar rats. (f) 2-DG (500 mg/Kg) was administered in control and exercised rats. Animals were immediately exposed to food for a 12-hour period (*n* = 12–15 animals per group). (g, h, i, j) Representative Western blots of five independent experiments showing hypothalamic lysates from Wistar rats. (k) Exercise decreases food intake in the fasting state (48 h fasting). Animals were immediately exposed to food for a 12-hour period (*n* = 12–15 animals per group). (l, m, n, o) Representative Western blots of five independent experiments showing hypothalamic lysates from Wistar rats. Phospho-AMPK^thr172^, threonine-phosphorylated AMPK and total AMPK; phospho-ACC^ser79^, serine phosphorylated ACC and total ACC; phospho-p70S6Kinase^thr389^, threonine phosphorylated p70S6Kinase and total p70S6K; phospho-4EBP1^thr70^, threonine phosphorylated 4EBP1 and total 4EBP1. Data are the means±SEM. * *p*<0.05, ** *p*<0.01, *vs.* control group; # *p*<0.05, ## *p*<0.001 *vs.* AICAR- or 2-DG-stimulated control group.

Consistent with food intake, AICAR increased AMPK threonine and ACC serine phosphorylation levels in the hypothalami of control rats, whilst in exercised animals, AICAR did not change AMPK/ACC phosphorylation status (Figures 3b and c). Comparing AICAR treated groups (control *vs.* exercise), exercised animals showed reductions in AMPK threonine and ACC serine phosphorylation of 52% and 31%, respectively. AICAR reduced p70S6K and 4EBP1 threonine phosphorylation levels in the hypothalamus of control and exercised rats. However, comparing AICAR treated groups (control *vs.* exercise), exercised animals showed increases in p70S6K and 4EBP1 threonine phosphorylation of 230% and 310%, respectively (Figures 3d and e). The αAMPK, ACC, p70S6K and 4EBP1 protein levels were not different between the groups (Figures 3b–e, lower panels). Similar results were observed after intraperitoneal treatment with 2-DG, another pharmacological activator of AMPK (Figure 3f–j).

To be sure that the experiments represent a physiological condition we measured food intake in control and exercised animals after fasting. In the control animals, prolonged fasting (48 hours) increased ∼35% of food intake during 12-hours of refeeding period compared to control group. However, in the fasted rats, acute exercise session prevented fasting-induced hyperphagic response (Figure 3k). Comparing fasting treated groups (control *vs.* exercise), exercised animals showed reductions in AMPK threonine and ACC serine phosphorylation of 65% and 41%, respectively (Figures 3l and m). Comparing fasting groups (control *vs.* exercise), exercised animals showed increases in p70S6K and 4EBP1 threonine phosphorylation of 261% and 240%, respectively (Figures 3n and o). The αAMPK, ACC, p70S6K and 4EBP1 protein levels were not different between the groups (Figures 3l–o, lower panels).

### Intracerebroventricular α-LA reduces food intake by modulating AMPK-mTOR hypothalamic phosphorylation levels to a greater extent in exercised animals

α-LA is an essential cofactor of mitochondrial respiratory enzymes and exerts potent anti-obesity effects by suppressing hypothalamic AMPK activity [34]. The effects of α-LA (3 µg) intracerebroventricular administration, or its vehicle, on food intake control were studied by measuring the 12-hour total food intake after an acute exercise bout. In exercised rats, α-LA (3 µg) reduced food intake by 86% while control group showed a reduction of 58%. Comparing α-LA treated groups (control *vs.* exercise), exercised animals showed a 64% reduction in 12-hour total food intake (Figure 4a).

**Figure 4:** α-LA effects on 12-h cumulative food intake and AMPK/mTOR signaling, in the hypothalami of control and exercised rats. (a) α-LA (3 µg) was administered in control and exercised rats. Animals were immediately exposed to food for a 12-hour period (*n* = 8–10 animals per group). (b, c, d, e) Representative Western blots of four independent experiments showing hypothalamic lysates from Wistar rats. Phospho-AMPK^thr172^, threonine-phosphorylated AMPK and total AMPK (b); phospho-ACC^ser79^, serine phosphorylated ACC and total ACC (c); phospho-p70S6Kinase^thr389^, threonine phosphorylated p70S6Kinase and total p70S6K (d); phospho-4EBP1^thr70^, threonine phosphorylated 4EBP1 and total 4EBP1 (e). Data are the means±SEM. * *p*<0.05, *vs.* control group; # *p*<0.05, *vs.* exercised non-stimulated group.

To determine the effects of exercise on the AMPK-mTOR signaling pathway, α-LA was i.c.v. administered and AMPK, ACC, p70S6K and 4EBP1 phosphorylation levels were assessed in the hypothalamus of all rats. α-LA reduced AMPK and ACC phosphorylation levels, in the hypothalami of control and exercised rats. Comparing α-LA treated groups (control *vs.* exercise), in exercised animals α-LA reduced both AMPK threonine phosphorylation and ACC serine phosphorylation of 39% and 57%, respectively (Figures 4b and c).

α-LA induced p70S6K and 4EBP1 threonine phosphorylation in the hypothalami of control and exercised rats. Comparing α-LA treated groups (control *vs.* exercise), in exercised animals, α-LA increased p70S6K and 4EBP1 threonine phosphorylation of 19% and 11%, respectively (Figures 4d and e). α-LA did not change αAMPK, ACC, p70S6K and 4EBP1 protein expression (Figures 4b–e, lower panels).

### Intracerebroventricular leptin reduces food intake by modulating AMPK-mTOR hypothalamic phosphorylation levels to a greater extent in exercised animals

The effects of leptin (10^−6^ M) i.c.v. administration or its vehicle on food intake control were studied by measuring the 12-hour total food intake after an acute exercise bout. In exercised rats, leptin (10^−6^ M) reduced food intake by 43%, when compared with exercised plus vehicle treated group, while the control group showed a reduction of 25%, when compared with vehicle treated group. Comparing leptin-treated groups (control *vs.* exercise), exercised animals showed a 31% reduction in 12-hour total food intake (Figure 5a).

**Figure 5:** Leptin effects on 12-h cumulative food intake and AMPK/mTOR signaling, in the hypothalami of control and exercised rats. (a) Leptin (10^−6^ M) was administered in control and exercised rats. Animals were immediately exposed to food for a 12-hour period (*n* = 12–15 animals per group). (b, c, d, e) Representative Western blots of five independent experiments showing hypothalamic lysates from Wistar rats. Phospho-AMPK^thr172^, threonine-phosphorylated AMPK and total AMPK (b); phospho-ACC^ser79^, serine phosphorylated ACC and total ACC (c); phospho-p70S6Kinase^thr389^, threonine phosphorylated p70S6Kinase and total p70S6K (d); phospho-4EBP1^thr70^, threonine phosphorylated 4EBP1 and total 4EBP1 (e). Data are the means±SEM. * *p*<0.05, ** *p*<0.01, *vs.* control group; # *p*<0.05, ## *p*<0.01 *vs.* leptin-stimulated control group.

To determine the effects of exercise on AMPK-mTOR signaling pathway, leptin was i.c.v. administered and AMPK, ACC, p70S6K and 4EBP1 phosphorylation levels were assessed in the hypothalamus of all rats. Leptin reduced AMPK and ACC phosphorylation levels in the hypothalami of control and exercised rats. Comparing leptin-treated groups (control *vs.* exercise), in exercised animals, leptin reduced both AMPK threonine phosphorylation and ACC serine phosphorylation of 57% and 45%, respectively (Figures 5b and c). Leptin induced p70S6K and 4EBP1 threonine phosphorylation in the hypothalamus of control and exercised rats. Comparing leptin treated groups (control *vs.* exercise), in exercised animals, leptin increased both p70S6K and 4EBP1 threonine phosphorylation of 30% and 40% respectively (Figures 5d and e). The αAMPK, ACC, p70S6K and 4EBP1 protein levels were not different between the groups (Figures 5b–e, lower panels).

### Role of IL-6 in anorectic response to leptin

Hypothalamic IL-6 expression was detected in control animals; however, a 420% increase was observed in the exercised group (Figure 6a). We tested whether the inhibitory effects of leptin on food intake depends on IL-6, by i.c.v. infusion of anti–IL-6 antibody into exercised rats. Treatment with leptin (10^−6^ M) markedly reduced 12-h food intake in exercised rats pretreated with vehicle, although pretreatment with anti–IL-6 antibody blocked exercise-induced leptin responsiveness in a concentration-dependent manner (Figure 6b).

**Figure 6:** Blockade of leptin induced inhibition of food intake by anti–IL-6 antibody. Hypothalami from rats were prepared as described in *Research Design and Methods*. (a) Tissue extracts from control and exercised rats were immunoblotted with anti–IL-6 antibody. (b) Leptin was injected intracerebroventricularly in control rats, exercised rats and exercised rats pretreated with anti–IL-6 at the doses indicated, and the animals were immediately exposed to food for a 12-hour period (*n* = 10–12 animals per group). (c, d, e, f) Representative Western blots of four independent experiments showing hypothalamic lysates from Wistar rats. Phospho-AMPK^thr172^, threonine-phosphorylated AMPK and total AMPK (c); phospho-ACC^ser79^, serine phosphorylated ACC and total ACC (d); phospho-p70S6Kinase^thr389^, threonine phosphorylated p70S6Kinase and total p70S6K (e); phospho-4EBP1^thr70^, threonine phosphorylated 4EBP1 and total 4EBP1 (f). Data are the means±SEM. *p<0.05, vs. control, **p<0.05, vs. control plus leptin, #*p*<0.05, *vs.* exercise plus leptin.

Both AMPK and ACC phosphorylation levels, reduced by exercise, were reversed by anti–IL-6 antibody (Figure 6c and d). We also observed that the increased phosphorylations of p70S6K and 4EBP1, induced by exercise, were also reversed by anti–IL-6 infusion (Figures 6e and f). The αAMPK, ACC, p70S6K and 4EBP1 protein levels were not different between the groups (Figures 6c–f, lower panels).

### The role of IL-6 on leptin responsiveness in the hypothalamus of diet-induced obesity (DIO) rats

We next investigated the effect of IL-6 on leptin responsiveness in the hypothalamus of diet-induced obesity (DIO) rats after acute exercise. Hypothalamic IL-6 expression was detected in the hypothalamus of diet-induced obesity (DIO) rats; however, a 156% increase was observed in the DIO rats after acute exercise (Figure 7a). The effects of leptin (10^−6^ M) i.c.v. administration on energy intake control were studied by measuring the 12-hour total food intake after an acute exercise bout in DIO rats. Comparing leptin-treated rats (control vs. DIO), the energy intake was 28% higher in DIO rats after leptin infusion. However, the i.c.v. infusion of leptin was able to reduce the energy intake by about 31% in DIO rats after the exercise protocol, compared to DIO rats at rest (Figure 7b). Interestingly, the i.c.v. pretreatment with anti-IL-6 antibody (25 ng) blunted the anorexigenic effects of leptin in exercised DIO rats.

**Figure 7:** Leptin effects on 12-h cumulative food intake and AMPK/mTOR signaling in the hypothalami of control, DIO and exercised DIO rats. (a) Representative Western blots of five independent experiments showing hypothalamic IL-6 expression in DIO Wistar rats at rest and immediately after acute exercise. (b) Leptin (10^−6^ M) was administered in control, DIO and exercised DIO rats. Animals were immediately exposed to food for a 12-hour period (*n* = 12–15 animals per group). (c, d, e and f) Representative Western blots of five independent experiments showing hypothalamic lysates from Wistar rats. Phospho-AMPK^thr172^, threonine-phosphorylated AMPK and total AMPK (c); phospho-ACC^ser79^, serine phosphorylated ACC and total ACC (d); phospho-p70S6Kinase^thr389^, threonine phosphorylated p70S6Kinase and total p70S6K (e); phospho-4EBP1^thr70^, threonine phosphorylated 4EBP1 and total 4EBP1 (f). Data are the means±SEM. * *p*<0.05, *vs.* control group, # *p*<0.05, *vs.* DIO group.

To determine the effects of exercise on the AMPK-mTOR signaling pathway in the hypothalamus of DIO rats, leptin was i.c.v. administered and AMPK, ACC, p70S6K and 4EBP1 phosphorylation levels were assessed in the hypothalamus. The suppressive effects of i.c.v. infusion of leptin on AMPK and ACC phosphorylation were impaired in the hypothalamus of DIO rats by about 58 and 54%, respectively, when compared to the control group (Figure 7c and d). In exercised DIO rats, leptin reduced the phosphorylation of AMPK by 65% and ACC by 37%, compared to DIO rats at rest and the i.c.v. pretreatment with anti-IL6 antibody before the exercise protocol, reversed the suppressive effects of leptin on AMPK/ACC pathway in the hypothalamus of exercised DIO rats (Figures 7c and d). The AMPK and ACC protein levels did not differ between the groups (Figures 7c and d, lower panels).

In addition, p70S6K and 4EBP1 phosphorylation in the hypothalamus of DIO rats after i.c.v. leptin infusion was reduced by about 46% and 45%, respectively, when compared to the control group. In exercised DIO animals, leptin increased the phosphorylation of p70S6K by 62% and 4EBP1 by 59%, compared to DIO rats at rest. I.c.v. pretreatment with anti-IL6 antibody before the exercise protocol blocked these effects in the hypothalamus of exercised DIO rats (Figures 7e and f). The p70S6K and 4EBP1 protein levels were not different between the groups (Figures 7e and f, lower panels).

### Blocking effects of AICAR and Rapamycin on leptin-induced anorexia

We tested whether the i.c.v. administration of AICAR or Rapamycin, 60 minutes before the administration of leptin (10^−6^ M), prevents the anorexigenic effects of leptin. Leptin (10^−6^ M) treatment markedly reduced 12-h food intake in both control and exercised groups, although leptin was much more effective in exercised rats. AICAR (0.5 mM) or Rapamycin (25 µg), at doses that do not alter ingestion, completely blocked the suppression of food intake induced by an i.c.v. injection of leptin (10^−6^ M) (Figure 8a). The i.c.v. administration of leptin (10^−6^ M) to exercised rats pretreated with vehicle reduced AMPK and ACC phosphorylation in the hypothalamus by 63% and 60% respectively, compared with the control group. The administration of AICAR increased AMPK threonine and ACC serine phosphorylation, although at this dose, AICAR was not sufficient to induce significant an increase in food intake in exercised animals (data not shown). Comparing exercised animals, i.c.v. administration of leptin (10^−6^ M) to rats pretreated with AICAR increased both AMPK and ACC phosphorylation levels in the hypothalamus (Figures 8b and c).

**Figure 8:** Blocking effects of AICAR and Rapamycin on leptin-induced anorexia. (a) Effect of i.c.v. administration of leptin on exercised rats; pretreatment with AICAR or Rapamycin (*n* = 8–10 animals per group). (b, c, d, e) Representative Western blots of five independent experiments showing hypothalamic lysates from Wistar rats. Phospho-AMPK^thr172^, threonine-phosphorylated AMPK and total AMPK (b); phospho-ACC^ser79^, serine phosphorylated ACC and total ACC (c); phospho-p70S6Kinase^thr389^, threonine phosphorylated p70S6Kinase and total p70S6K (d); phospho-4EBP1^thr70^, threonine phosphorylated 4EBP1 and total 4EBP1 (e). Data are the means±SEM. *p<0.05, *vs.* other groups.

The i.c.v. administration of leptin (10^−6^ M) to exercised rats pretreated with vehicle induced p70S6K and 4EBP1 phosphorylation in the hypothalamus of 60% and 70%, respectively, compared with the control group. Comparing exercised animals, i.c.v. administration of leptin (10^−6^ M) to rats pretreated with AICAR reduced both p70S6K and 4EBP1 phosphorylation levels in the hypothalamus. Exercised animals pretreated with Rapamycin also reduced hypothalamic p70S6K and 4EBP1 phosphorylation (Figures 8d and e). The αAMPK, ACC, p70S6K and 4EBP1 protein levels were not different between the groups (Figures 8b–e, lower panels).

## Discussion

During the last decade, a substantial number of studies have investigated the role of physical activity in the control of energy intake in rodents [5], [6], [35] and in humans [36]–[38]. However, the molecular mechanisms by which exercise controls food intake are still unsolved. Several experimental studies have demonstrated that neither acute [5], [36] nor chronic [6], [39] exercise per se change food intake, on the other hand, accumulating evidence shows that both acute and chronic exercise potentiate the anorexigenic effects of leptin in the hypothalamus. Our data indicate that IL-6 signaling through AMPK and mTOR reduces food intake in a dose-dependent manner. Leptin, as well as α-LA infusion, reduced food intake in exercised rats to a greater extent than that observed in control animals. Conversely, AICAR, 2-DG and fasting increased food intake in exercised rats to a lower extent than that observed in control animals. Exercise was associated with the effects of leptin on the AMPK/mTOR pathway activity in the hypothalamus. In addition, we investigated the regulatory role of IL-6 in mediating the increase in leptin responsiveness in the hypothalamus. Treatment with leptin markedly reduced food intake, AMPK activity and increased mTOR activity in exercised rats that were pretreated with vehicle, although no increase in response to leptin-induced anorexia and modulation of AMPK/mTOR pathway were detected after i.c.v. pretreatment with anti-IL-6 antibody. Taken together, these results suggest that IL-6 is a major component of the effects of exercise on the control of food intake.

Increasing evidence shows that leptin and IL-6 activates AMPK in the peripheral tissues, such as skeletal muscle and adipose tissue, increasing fatty acid oxidation and glucose uptake in these tissues [40]–[42], however, leptin has an opposing effect in hypothalamic tissue, reducing neuronal AMPK activity [12], [43]. As well as in response to leptin, in the present study, we demonstrated that IL-6 alone reduced AMPK phosphorylation in the hypothalamus of rats. We also show that, IL-6 increased ATP levels and decreased the AMP/ATP ratio in the hypothalamus (figures 1b–d), but the mechanisms by which IL-6 modulates the ATP levels require further investigations.

A number of recent studies have shown that AMPK plays a key role in regulating both energy intake and expenditure [12], [34], [44], [45]. In peripheral tissues, such as skeletal muscle, activation of AMPK switches on energy producing pathways and switches off energy consuming pathways. In the hypothalamus, activation of AMPK leads to increased feeding, thereby increasing energy intake. Conversely, inhibition of AMPK in the hypothalamus reduces food intake. These dual functions of AMPK suggest that it may act to coordinate energy expenditure with energy intake. There is already some evidence that this may be the case in one situation. More recently, Gao and colleagues [10] demonstrated that the hypothalamic ACC activation makes an important contribution to the anorexigenic effects of leptin that are mediated by AMPK. The aim of this study was to investigate whether IL-6 could affect AMPK activity in the hypothalamus, thereby providing a potential mechanism for the coordination of energy expenditure and energy intake during, or following exercise. Beyond STAT3 activation, we detected changes in the hypothalamic AMPK activity in rats after i.c.v. infusion of IL-6; we show that, IL-6 markedly decreased phospho-AMPK abundance (an index of activity) in the hypothalamus. In accordance with the reduction in AMPK^thr172^ phosphorylation, we observed that, after IL-6 administration, hypothalamic AMP∶ATP ratio was decreased.

Wallenius et al [28] elegantly showed that long-term peripheral IL-6 treatment to Il6^−/−^ mice caused a decrease in body weight. In addition to increasing energy expenditure, IL-6 may prevent obesity by inhibiting feeding as obese IL-6^−/−^ mice had increased absolute food intake. However, central IL-6 treatment at the same dose that we used does not influence food intake in mice. In concordance with our results another study of the same group showed a reduced daily food intake over a two-week ICV treatment period with IL-6 in rats indicating a different pattern of response between rats and mice [46].

The mTOR, an evolutionary conserved serine-threonine kinase, central to integrating similar signals to control food intake, has now emerged as a detector of hormonal and nutritional signals in the hypothalamus [13], [15]. In this study, we investigated whether IL-6 activates mTOR. IL-6 increased mTOR activity; moreover inhibition of central mTOR reversed the anorectic effect of IL-6. In addition, the anorexigenic effect of IL-6 was absent in AICAR- and Rapamycin-pretreated rats, however, pretreatment with LY294002 - a PI(3)K inhibitor - had no effect on IL-6 induced anorexia, indicating that, in the hypothalamus, the effect of IL-6 is independent of the PI(3)K pathway. Signaling through gp130 commonly results in activation of PI(3)K, and IL-6 can activate PI(3)K [47] and its downstream target Akt [48]–[51], but it should be noted that this effect has not been observed in all studies [52], suggesting a tissue-dependent effect.

Next, we investigated whether the increased sensitivity of the leptin action on food intake induced by exercise, could be due to the modulation of AMPK activity. As previously shown [43], exercise, per se, does not alter AMPK activity in the hypothalamus; however, we observed that the normal inhibition of AMPK phosphorylation and activity in the hypothalamus, induced by leptin administration, was improved in both lean and diet-induced obesity rats after acute protocol of exercise.

In addition, we did not observe any normal stimulation of AMPK activity by AICAR in the hypothalamus of exercised rats, indicating that AMPK pathway is disrupted. This observation agrees with data from aging studies in which acute stimulation with AICAR was blunted in skeletal muscle of old rats [53]. Furthermore, fasting and the use of another activator of AMPK (2-DG) in exercising rats resulted in a lower activation of AMPK when compared to the control animals. In contrast, the pharmacological inhibition of AMPK by α-LA results in a greater inhibition of AMPK activity, compared to control animals.

The mechanism by which exercise inhibits AMPK-induced food intake in the hypothalamus is not clear. Several lines of evidence point to a possible link between inhibited AMPK-induced food intake in the hypothalamus and IL-6 signaling through the AMPK/mTOR pathway. Firstly, we found that the leptin-inhibited food intake enhanced by exercise was blunted by anti-IL-6 antibody. Secondly, exercise induced increased response of leptin-inhibited AMPK signaling was reverted by AICAR. Finally, exercise induced increased responsiveness of leptin stimulated mTOR signaling was reverted by rapamycin.

Our data are in accordance with earlier studies demonstrating that IL-6 treatment enhances energy expenditure in both rodents and humans [28], [54]–[56]. In exercising rats, hypothalamic leptin and insulin responsiveness are increased in an IL-6-dependent manner [5], [6]. It has been previously shown that IL-6 treatment stimulates energy expenditure at the level of the brain in rodents [28], [55], [57], and it might be assumed that endogenous IL-6 also acts on the brain during exercise. The IL-6 exerting this effect during exercise could be produced by the brain itself, which has been shown to have increased IL-6 production during exercise [58]. Alternatively, the large quantities of endocrine IL-6 produced from working skeletal muscle [58] might reach appropriate sites in the brain [21], [59], [60].

Interestingly, we did not observe any difference in food intake over a 12-h period, although the levels of hypothalamic IL-6 dramatically increased after exercise. At first glance, these data appear to be contradictory. However, a large decrease in insulin level was observed after exercise, and we have previously shown a synergic effect of IL-6 on the insulin and leptin signaling pathway, in the rat hypothalamus [5]. Since we did not observe modifications in the phosphorylation of JAK2 and the downstream targets of mTOR after exercise, these data suggest that the cross-talk between insulin, IL-6 and leptin have an essential role in controlling food intake after exercise. In this case, it is possible that increases in IL-6 levels were counterbalanced by the reduction in insulin levels.

However, the present study has certain limitations. Exercise per se did not evoke any meaningful effect in terms of food intake; rather, it seemed to enhance the anorectic effect of exogenous leptin. Thus, the data presented herein may suggest but do not establish the mechanism by which long term exercise decreases leptin levels; whilst increases the response to leptin, contributing to its food-suppressive actions. Furthermore, settings of activation of AMPK or inactivation of mTOR were selected to induce changes in target protein phosphorylation, but not food intake. Such dissociation does not preclude a pharmacological rather than physiological effect of our data.

Increased responsiveness of leptin action in the hypothalamus, through modulation of the AMPK-mediated pathway by exercise, could be pathophysiologically important in the prevention of obesity. Recent studies have shown that modulation of leptin signaling through the AMPK pathway could be involved in the development of obesity [61]. Taken together, these data indicate that the anti-obesity actions, induced by leptin, could be increased due to the more pronounced inhibition of the AMPK pathway observed after leptin infusion in the hypothalamus of both lean and diet-induced obesity rats after acute exercise. If the mechanism used by IL-6 to reduce food intake is AMPK-dependent, as our results suggest, the defective activation of AMPK in the hypothalamic neurons induced by exercise may increase the ability of leptin to reduce food intake.

In conclusion, exercise improved the AMPK and mTOR responses to leptin administration and contributed to appetite-suppressive actions. This increased dynamic responsiveness of the AMPK/mTOR pathway to leptin could provide information regarding the molecular mechanism underlying the biological sensitivity to leptin in exercise. Furthermore, these findings provide support to the hypothesis that AMPK and mTOR interact in the hypothalamus to control feeding in exercised rats, in an IL-6-dependent manner.

## Methods

### Antibodies and Chemicals

Reagents for SDS-polyacrylamide gel electrophoresis and immunoblotting were from Bio-Rad (Richmond, CA, USA). Tris[hydroxymethyl]amino-methane (Tris), aprotinin, ATP, dithiothreitol, phenylmethylsulfonyl fluoride, Triton X-100, Tween 20, glycerol, and bovine serum albumin (fraction V) were from Sigma Aldrich (St. Louis, MO, USA). Protein A-Sepharose 6 MB and Nitrocellulose paper (Hybond ECL, 0.45 µm) from Amersham Pharmacia Biotech United Kingdom Ltd. (Buckinghamshire, United Kingdom). Ketamin was from Parke-Davis (São Paulo, SP, Brazil) and diazepam and thiopethal were from Cristália (Itapira, SP, Brazil). Anti-phospho-[Ser^79^] ACC (rabbit polyclonal, #07-184) and anti-phospho- [Tyr^1007/1008^] JAK2 (rabbit polyclonal, AB3805) antibodies were from Upstate Biotechnology (Charlottesville, VA, USA). Anti-ACC (goat polyclonal, sc-26816), anti-JAK2 (rabbit polyclonal, sc 278), anti-STAT3 (rabbit polyclonal, sc 483) and anti-IL-6 (rabbit polyclonal, sc-7920) antibodies were from Santa Cruz Biotechnology, Inc. Anti-phospho-[Thr^172^] AMPKα (rabbit polyclonal, #2531), anti-AMPKα (rabbit polyclonal, #2532), anti-phospho- [tyr705] STAT3 (rabbit polyclonal, #9135), anti-phospho- [Thr389] p70S6K (rabbit polyclonal, #9205), anti-p70S6K (rabbit polyclonal, #9202), anti-phospho- [Thr70]4EBP1 (rabbit polyclonal, #9455), anti-4EBP1 (rabbit polyclonal, #9452), anti-phospho- [Ser 473]Akt (rabbit polyclonal, #9271), and anti-Akt (rabbit polyclonal, #9272) were from Cell Signalling Technology (Beverly, MA, USA). Leptin, LY294002, and Interleukin-6 were from Calbiochem (San Diego, CA, USA); 5-Aminoimidazole-4-carboxamide 1-β-D-ribofuranoside (AICAR), 2-Deoxy-D-glucose and α-lipoic acid were from Sigma Chemical Co. (St. Louis, MO). Rapamycin was from LC Laboratories (Woburn, MA, USA). Routine reagents were purchased from Sigma Chemical Co. (St. Louis, MO) unless otherwise specified.

### Serum insulin and leptin quantification

Plasma was separated by centrifugation (1100 *g*) for 15 minutes at 4°C and stored at −80°C until assayed. RIA was employed to measure serum insulin, according to a previous description [62]. Leptin concentrations were determined using a commercially available Enzyme Linked Immuno Sorbent Assay (ELISA) kit (Crystal Chem Inc, Chicago, IL).

### Experimental Animals

Male Wistar rats (8 weeks old/250–300 g) obtained from the University of Campinas Animal Breeding Center were used in the experiments. The investigation was approved by the ethics committee and followed the University guidelines for the use of animals in experimental studies and conforms to the *Guide for the Care and Use of Laboratory Animals*, published by the US National Institutes of Health (NIH publication no. 85-23 revised 1996). The animals were maintained on 12h∶12h artificial light–dark cycles and housed in individual cages.

### Diet induced obesity (DIO)

Male 4-wk-old Wistar rats from the University of Campinas Breeding Center were randomly divided into two groups, control, fed standard rodent chow (3948 kcal.Kg^−1^) and DIO, fed a fat-rich chow (5358 kcal.Kg^−1^) *ad libitum* for 3 months and then submitted to the different experimental protocols. This diet composition has been previously used [63].

### Intracerebroventricular (i.c.v.) cannulation

The animals were stereotaxically instrumented under intraperitoneal injection of a mix of ketamin (10 mg) and diazepam (0.07 mg) (0.2 ml/100 g body weight) with a chronic 26-gauge stainless steel indwelling guide cannula, aseptically placed into the third ventricle (0.5 mm posterior and 8.5 mm ventral to bregma), as previously described [64]. After a 1-wk recovery period, cannula placement was confirmed by a positive drinking response after administration of Angiotensin II (40 ng/2 µL); animals that did not drink 5 mL of water within 15 minutes after treatment were not included in the experiment.

### Exercise Protocol

Rats were acclimated to swimming for 2 days (10 min per day). On the day of the experiment, animals swam in groups of four, in plastic barrels of 45 cm in diameter, filled to a depth of 50 cm. Water temperature was maintained at 34–35°C. They performed two 3-h exercise bouts, separated by one 45-min rest period, as previously described [65]. After the last exercise bout, some rats were injected into the cannula and food intake was determined over the next 4 and/or 12 h; the other rats were injected into the cannula and then anesthetized with intraperitoneal injection of sodium thiopethal (5 mg/100 g body weight) and hypothalamus was removed.

### Treatments

For acute treatments, rats were deprived of food for 6 h with free access to water and i.p. injected (200 µl bolus injection) with either vehicle or 2-DG (500 mg/kg) or i.c.v. injected (3 µl bolus injection) with either vehicle, IL-6 (100 ng or 200 ng), AICAR (0.5 or 2.0 mM), Rapamycin (25 µg), α-LA (3 µg), leptin (10^−6^ M), LY294002 (50 µM) or anti-IL-6 antibody. Similar studies were carried out in rats that were initially pre-treated with i.c.v. microinjection of vehicle, AICAR, Rapamycin, anti-IL-6 antibody or LY294002, and after 60 min with i.c.v. microinjection of IL-6 or leptin. Thereafter, standard chow was given and food intake was determined by measuring the difference between the weight of chow given and the weight of chow at the end of 4 and/or 12-h periods. All acute treatments were performed at 5:00 and 6:00 p.m.

### Western Blot Analysis

After exercise and i.c.v. treatments, rats were anaesthetized with intraperitoneal injection of a mix of ketamin (10 mg) and diazepam (0.07 mg) (0.2 ml/100 g body weight), and used as soon as anesthesia was assured by the loss of pedal and corneal reflexes. The rats were killed, and hypothalamus was quickly removed, minced coarsely and homogenized immediately in a freshly prepared ice-cold buffer (1% Triton X-100, 100 mmol/l Tris pH 7.4, 100 mmol/l sodium pyrophosphate, 100 mmol/l sodium fluoride, 10 mmol/l EDTA, 10 mmol/l sodium vanadate, 2 mmol/l phenyl methylsulphonyl fluoride and 0.1 mg aprotinin) suitable for preserving phosphorylation states of enzymes and Western blot was performed, as previously described [66]. Insoluble material was removed by centrifugation (50 000 g) for 25 minutes at 4°C. Total extracts of hypothalamus were prepared and 0.25 mg total proteins were separed by SDS-PAGE. After SDS-PAGE (15% resolving gels for phospho-4EBP1 and 4EBP1; 12% resolving gels for phospho-AMPK, AMPKα2; phospho-p70S6K, p70S6K, phospho-Akt, Akt, phospho-STAT3 and STAT3; 8% resolving gels for phosphor-JAK2 and JAK2; 6.5% resolving gels for ACC and phospho-ACC), proteins were transferred from gel to nitrocellulose membrane. Membranes were blocked in 5% nonfat dried milk in PBST (139 mM NaCl, 2.7 mM KH_2_PO_4_, 9.9 mM Na_2_HPO_4_, and 0.1% Tween 20) for 2 hours and then incubated overnight with specific antibodies. After incubation with the relative second antibody, immune complexes were detected using the ECL method. Results were visualized by autoradiography using preflashed Kodak XAR film (Eastman Kodak, Rochester, N.Y., USA) with Cronex Lightning Plus intensifying screens at −80°C for 12–48 h. (Mass., USA). Band intensities were quantified by optical densitometry of developed autoradiographs (Scion Image software - *Scion Corporation*, Frederick, Md., USA).

### Confocal microscopy

Paraformaldehyde-fixed hypothalami were sectioned (5 µm). The sections were obtained from hypothalamus of six rats per group in the same localization (antero-posterior = −1.78 from bregma) and used in regular single- or double-immunofluorescence staining using DAPI, anti-IL6 receptor (IL6R), anti-AMPK, anti-phospho-p70S6K (1∶200; Santa Cruz Biotechnology), antibodies, according to a previously described protocol [67]. Analysis and photodocumentation of results were performed using a LSM 510 laser confocal microscope (Zeiss, Jena, Germany). The anatomical correlations were made according to the landmarks given in a stereotaxic atlas [68].

### Chromatography

After exercise, i.c.v. infusion of IL-6 or vehicle, rats were anaesthetized, and used as soon as anesthesia was assured by the loss of pedal and corneal reflexes. The animals were killed and, within 40 seconds, the cranium was opened, the brain was removed and the hypothalamus was quickly dissected and frozen in liquid N_2_ for chromatographic analyses.

Chromatographic analyses were carried out on a Waters Alliance equipment series 2695 (Milford, MA, USA) equipped with a quaternary pump, an autosampler, a degasser, and a Waters 2475 fluorescence detector model. The fluorescence of derivatized compounds (ATP, ADP, AMP, and ADO) was monitored with excitation and emission wavelengths set at 280 and 420 nm, respectively. Chromatographic separations of the compounds were achieved at room temperature, using a reversed-phase Cosmosil 5C18-MS column (150×4.6 mm i.d.; 5 µm particle size) with a Cosmosil guard column (5C18-MS 10×4.6 mm) purchased from Phenomenex (Torrance, CA, USA). The mobile phase composition was 50 mmol/L KH_2_PO_4_, 25 mmol/L citric acid (pH 4.5), and methanol (90∶10, v/v), which was prepared immediately before use and filtered through a 0.45 µm filter (Millipore, Milford, MA, USA). The column was equilibrated and eluted under isocratic conditions using a flow rate of 1.0 ml/min. The chromatographic run time for each analysis was 20 min. Aliquots of 25 µl were injected into the HPLC system. System control, data acquisition, and processing were performed with a PC-Pentium IV Processor personal computer from Dell, operated with Microsoft Windows XP version 2003 and Waters Empower 2002 chromatography software. A validation chromatographic run included a set of calibration samples assayed in duplicate and quality control samples at four levels in triplicate. The standard calibration curves for known amounts of ATP, ranging from 0.025 to 10.0 µmol/L, were linear (R>0.999) and could be described by the linear regression equation: *y* = 0.4992*x−0.0463 (*n* = 4, *P*<0.0001, *r* = 0.9997), in which *y* is the ATP concentration in micromoles and *x* is the chromatogram peak area.

### Statistical Analysis

All numeric results are expressed as the means±SEM of the indicated number of experiments. The results of blots are presented as direct comparisons of bands or spots in autoradiographs and quantified by optical densitometry (Scion Image). Statistical analysis was performed by employing the ANOVA test with *Bonferroni post test*. Significance was established at the *p*<0.05 level.
